RETRACTED

# Electrophysiological Characteristics of Cervical Spinal Stenosis

**DOI:** 10.1155/2022/7522664

**Published:** 2022-06-26

**Authors:** Yanrong Wang, Yinping Zhan, Xiaolan Jin, Dandan Shen, Ling Wang, Tingting Cao, Hong Jiang

**Affiliations:** Department of Electromyography, Zhejiang University School of Medicine Sir Run Run Shaw Hospital, Hangzhou, China

## Abstract

**Objective:**

To investigate electrophysiological characteristics of patients with cervical spinal stenosis (CSS) due to cervical disc herniation.

**Methods:**

A total of 51 patients with CSS diagnosed in our hospital from January 2018 to March 2020 were selected. According to magnetic resonance imaging (MRI), the degree of spinal cord compression was divided into 1-3 grades, namely, group A (MRI grade 1), group B (MRI grade 2), and group C (MRI grade 3), with 17 cases in each group. Subsequently, we analyzed the correlation of the degree of spinal cord compression with the general information, clinical data, and electromyography (EMG) of patients.

**Results:**

Compared with group A and group B, group C had the longest disease course [(48.06 ± 17.71) months], the lowest JOA score (4.59 ± 2.15), and the highest number of positive results of EMG (EMG: A/B/C, 25/51/77); there were significant differences among the 3 groups. And group C had the higher number of positive cases of both upper and lower limbs in SEP test compared with the other two groups (SEP: A/B/C: 12/18/29: *χ*^2^ = 7.559, *P* = 0.023). According to correlation analysis, MRI grading had no association with gender, age, and spinal canal diameter/volume but was positively correlated with disease course and negatively correlated with JOA score.

**Conclusion:**

This study primarily verifies that higher MRI grade of CSS is associated with longer disease duration and lower JOA score and EMG. The obtained results secondarily demonstrate the correlation between abnormal neurological status and the MRI grade.

## 1. Introduction

Cervical spinal stenosis (CSS) can be caused by cervical disc herniation, tumors, fractures, and other factors. This disease causes damage to motor neurons and patients with limb numbness and weakness and bladder and bowel dysfunction [1–3]. Such symptoms, which seriously affect the quality of life of patients, can be relieved by physiotherapy, immobilization, or other treatment methods. However, surgical treatment is advocated for patients with rapid development of spinal cord invasion. Imaging examination is relied for the diagnosis and the choice of surgical approach. X-ray can visually display the standard lateral sagittal diameter of the cervical spinal canal, but it fails to provide accurate information about the soft tissue. By contrast, computed tomography (CT) and magnetic resonance imaging (MRI) are generally considered to be sensitive in the detection of CSS. CT can clearly reveal the shape of the cervical spinal canal and the degree of stenosis, but combined application of CT and other radiology modalities is necessary for the assessment of CSS due to the unsatisfactory CT imaging result of the spinal canal soft tissues; MRI can accurately reflect the longitudinal dura mater and spinal cord compression state, but its assessment of the lesion and physiological bone structure is poor [4–10].

RETRACTED

The number of patients with CSS in China has continued to increase year by year. Although the morphological changes of the bone structure, nerve roots, and spinal cord of patients can be understood through CT and MRI, the evaluation of neurological function is still insufficient. Nerve electrophysiology can serve as a supplement to radiology modalities. For example, electromyography (EMG) shows values in diagnosing lesions ofperipheral nerve, and muscles, especially for abnormalities of lower motor neurons, nerve root, nerve plexus, neuromuscular junction, and muscles. EMG also can help differentiate the nature, location (nerve roots, plexus, or peripheral nerve), and severity of lesions to assist in correct clinical diagnosis and selection of treatment options. And diseases unsuitable for surgery can be excluded after EMG, such as motor neuron disease, peripheral neuropathy, and other neurological diseases [11, 12].

Currently, the relationship between neurological function and the degree of spinal canal compression is not clear. In this study, the cases of CSS confirmed on MRI received nerve electrophysiology. Based on the examinations, we assessed the correlation between MRI grades and patients' general data and MRI grade and neurological dysfunction. The specific report is shown as follows.

## 2. Data and Methods

### 2.1. General Information of Patients

A total of 51 patients with CSS diagnosed in our hospital from January 2018 to March 2020 were selected. They were aged 18 to 75, with 33 males and 18 females. This study was approved by the Ethics Committee of Zhejiang University School of Medicine Sir Run Run Shaw Hospital (2022-0138).

Inclusion criteria are as follows: (1) MRI showed obvious CSS caused by bony narrow or backward protrusion or prolapse of intervertebral disc (Figure 1); (2) patients gave informed consent.

Exclusion criteria are as follows: (1) patients with cervical fracture and spinal tuberculosis (confirmed by MRI), (2) patients with a history of cervical spine surgery and tumor occupying, and (3) patients with suspected peripheral nerve injury and extensive nerve damage.

RETRACTED

### 2.2. MRI Grading and Nerve Electrophysiology

MRI grading was developed as the following criteria [13]: (1) grade 1: obliteration of subarachnoidale space >50%, without signs of cord deformity; (2) grade 2: central canal stenosis, without signs of cord deformity; (3) grade 3: spinal cord signal enhancement on T2-weighted image. Based on MRI grading, the 51 included patients were, respectively, divided into groups A, B, and C (17 cases/group) to increase the comparability between EMG and MRI grading.

Keypoint electromyographic instrument (Guangzhou Weidi Medical Instrument Co., Ltd.) was adopted. Specifically, with the ambient temperature >25, and skin temperature of patients >32, the patients sitting received NCV test and EMG. One upper limb with severe symptoms was detected firstly, and the other upper limb was detected subsequently in case of some abnormalities.

### 2.3. Observational Indicators

1. General information of patients: age, gender, disease duration, JOA score at admission [14], comorbidity, MRI grade, and spinal canal diameter/volume
2. EMG: muscles of upper limb; the first interosseous, Pronator teres, extensor digitorum communis, brachioradialis, triceps brachii and rhomboideus
3. Somatosensory evoked potential (SEP): SEPs of tibial nerve of both lower limbs and SEPs of median never of both upper limbs

Evaluation criteria of the above examinations were as follows [15]: (1) positive EMG: positive sharp wave, fibrillation wave, and high potential (amplitude ≥1.5 mv, duration ≥14 ms) of muscles; (2) positive nerve conduction: conduction velocity <45 of nerve of any upper limbs or conduction velocity <40 of nerve of any lower limbs; (3) positive SEP: amplitude <0.2*μ*v, bilateral amplitude ratio <50%, or bilateral latency difference ≥1.5 ms.

### 2.4. Statistical Analysis

SPSS 22.0 was applied for data processing. Measurement data were expressed as ($\bar{x}\pm s$), and *t*-test was performed for comparison among groups, while enumeration data were expressed as *n* or % and chi-square test was utilized for comparison between two groups. Spearman's correlation analysis was carried out. *P* < 0.05 represented a statistically significant test result.

## 3. Results

### 3.1. Analysis of the General Information of the Patients in Each Group

According to the comparison of general information of the patients, the following results were found. First, significant differences were observed among three groups in disease duration and JOA score; specifically, the longer the disease duration, the lower the JOA score. Besides, there was no significant difference in age, gender, comorbidity, and spinal canal diameter/volume (Table 1).

RETRACTED

### 3.2. Detection Results of EMG

Compared with the other two groups, group C also had significantly more positive cases in term of the first interosseous, pronator teres, brachioradialis, Extensor digitorum communis, triceps brachii and rhomboideus (all *P* < 0.05). This result suggested that higher MRI grade was associated with the higher number of EMG-positive cases (Table 2).

### 3.3. SEP Examination Results

Comparison of SEP results revealed that group C had the highest number of positive results (*n* = 29), followed by group A (*n* = 12), and group B (*n* = 18). It could be concluded that the higher MRI grade was associated with increased number of cases with positive SEP results and of cases with positive SEP results in both upper and lower limbs (A/B/C: 12/18/29: *χ*^2^ = 7.559, *P* =0.023, Table 3).

### 3.4. Correlation Analysis of MRI Grade and Information of Patients

MRI grade showed no correlation with gender, age, or spinal canal diameter/volume, but it was positively correlated with disease duration (*r* = 0.596, *P* ≤ 0.001) and negatively correlated with JOA score (*r* = −0.720, *P* ≤ 0.001). In other words, the higher the grade, the longer the disease duration and the lower the JOA score (Table 4).

## 4. Discussion

Clinical diagnosis of cervical spondylotic myelopathy mainly relies on CT, MRI, and other imaging examinations currently. However, some patients have different physical manifestations from the imaging results. For correct assessment and diagnosis, electrophysiology and cerebrospinal fluid examination can be effective technique to complement imaging [16, 17]. Some researches have shown that early stage of neurological impairment only accompanies with limb dysfunction, and the nerve electrophysiology examination data are normal in most of conditions [18]. As the disease progresses, axonal degeneration and demyelinating change occur and cause corresponding abnormalities in electrophysiological data, so clinicians often ignore such examination [18]. But some studies have reported that nerve electrophysiological examination can provide additional diagnostic information for CSS [19]. For example, EMG can reflect whether there is myogenic damage or neurogenic damage; SEP can observe lesions in the spinal cord, brainstem, thalamus, or sensory cortex of the brain. Additionally, nerve electrophysiological testing contributes to predicting the surgical outcome for patients requiring surgery, especially helpful for high-risk spinal cord injury surgery.

The degree of spinal cord compression and CSS grade show a significant positive correlation, but there are few reports on the relationship between the grade of CSS and nerve electrophysiology. Given this lack, we studied 51 patients with CSS. The results of this study indicated that, in group A (MRI grade 1), no abnormalities were found in EMG, and SEP of the patients, but some slightly physical dysfunctions still occurred. Besides, the JOA score was (10.24 ± 1.89), and the number of EMG and SEP positive cases was also small. The results of group A verified that early stage of neurological impairment only accompanied with limb dysfunction, and the electrophysiological examination data were normal. The quantity of positive cases of EMG, and SEP in group B (MRI grade 2) were significantly higher than those in group A, with the highest number of positive cases in group C. The above results suggested that the grade got higher and electrophysiological indicators changed. Specifically, the number of positive cases of EMG, and SEP increased, and that of positive cases of multiple nerves also increased, suggesting that with higher degree of spinal cord compression, nerve damage becomes more serious and more sites are damaged. Additionally, the MRI grade was not associated with gender, age, or spinal canal diameter/volume but positively correlated with disease duration and negatively with JOA score. So the longer the disease duration, the lower the JOA score and the higher the grade. The negative correlation between the grade and EMG indicators suggests that the higher MRI grade is correlated to a more severe nerve damage. Collectively, our primary conclusion is that higher MRI grade of CSS has a relationship with longer disease duration, lower JOA score, and more positive muscles of EMG. And our secondary finding is the association between abnormal neurological status and the MRI grade, which can act as clinical reference. However, this study has some limitations due to small sample size and the fact that patients were not selected completely at random.

RETRACTED

## 5. Conclusion

MRI grade of CSS is not associated with gender, age, and spinal canal diameter/volume. But it shows a positive correlation with disease duration and negative correlation with JOA score and EMG. Such correlations suggest that the higher the MRI grade, the longer the disease duration, the more positive muscles of EMG and the lower the JOA score.

## Figures and Tables

**Figure 1:** MRI shows obvious spinal stenosis caused by bony narrow or backward protrusion or prolapse of intervertebral disc.

**Table 1:** Analysis of the general information of the patients in each group.

Items	Group A (MRI grade 1, *n* = 17)	Group B (MRI grade 2, *n* = 17)	Group C (MRI grade 3, *n* = 17)	*F*/*χ*^2^	*P*
Age	59.65 ± 9.78	56.94 ± 10.23	57.47 ± 8.22	0.391	0.678
Gender	11/6	10/7	12/5	0.515	0.773
Disease duration	24.29 ± 7.95	34.18 ± 12.81	48.06 ± 17.71	13.440	≤0.001
JOA score	10.24 ± 1.89	7.65 ± 2.74	4.59 ± 2.15	25.972	≤0.001
Comorbidity (yes)	7	6	6	0.168	0.920
Spinal canal diameter/volume	0.27 ± 0.08	0.29 ± 0.08	0.26 ± 0.05	0.542	0.585

**Table 2:** Comparison of detection results of EMG (n).

EMG	Group A (*n* = 17)	Group B (*n* = 17)	Group C (*n* = 17)	*χ* ^2^	*P*
The first interosseous	3	7	13	12.037	0.002
Pronator teres	4	10	13	9.917	0.007
Brachioradialis	5	8	13	7.689	0.021
Extensor digitorum communis	3	5	11	8.724	0.013
Triceps brachii	5	10	13	7.761	0.021
Rhomboideus	5	11	14	10.200	0.006

**Table 3:** Comparison of detection results of SEP examination.

Items	Group A (MRI grade 1, *n* = 17)	Group B (MRI grade 2, *n* = 17)	Group C (MRI grade 3, *n* = 17)	*χ* ^2^	*P*
Median never of both upper limbs	6	8	13	6.139	0.046
Tibial nerve of both lower limbs	6	10	16	12.750	0.002
SEP (n, positive cases)	12	18	29	7.559	0.023

**Table 4:** Correlation analysis of MRI grade and information of patients.

Items	MRI grade	
	*r*	*P*
Age	-0.050	0.726
Spinal canal diameter/volume	-0.068	0.635
Disease duration	0.596	≤0.001
JOA score	-0.720	≤0.001

## Data Availability

The data used to support the findings of this study are available from the corresponding author upon request.
